The article "Cocreation from Emerging Opportunities: Occupational Therapists' Perspectives on Supporting Older Persons, in Japan" was published in 2022. Journal: Occup Ther Int.

# Cocreation from Emerging Opportunities: Occupational Therapists' Perspectives on Supporting Older Persons, in Japan

**DOI:** 10.1155/2022/5495055

**Published:** 2022-07-21

**Authors:** Peter Bontje, Staffan Josephsson, Yumi Tamura, Yu Ishibashi, Yuki Sakane, Yasuyo Horibe, Eric Asaba

**Affiliations:** ^1^Department of Neurobiology, Care Science and Society, Division of Occupational Therapy, Karolinska Institutet, Stockholm, Sweden; ^2^Graduate School of Human Health Sciences, Department of Occupational Therapy, Tokyo Metropolitan University, Tokyo, Japan; ^3^The Japanese Red Cross College of Nursing, DNGL (Disaster Nursing Global Leadership Program), Tokyo, Japan; ^4^Rehabilitation Department, Tango Central Hospital, Kyōtango, Japan; ^5^Aichi Medical College, Kiyosu, Japan; ^6^Stockholms Sjukhem, Unit for Research, Education, Development, and Innovation, Stockholm, Sweden

## Abstract

**Introduction:**

Practices of occupational therapists, particularly those supporting older persons with physical impairments, remain overly focused on remediating impairments, and implementation of occupation-centered practices remains fraught with difficulties. In Japan, this issue exists across the continuum from acute care to rehabilitation settings and into the community. This is despite the existence of international models and frameworks that place occupation at the core of the profession. Accordingly, there is a need to better understand how occupational therapists respond to the call for occupation-centered practices across the said continuum of care with this population. The aim of this study was at exploring and understanding occupational therapists' experiences of supporting the resumption of occupations among older persons with physical impairments, in Japan.

**Methods:**

Embedded in a constructivist world view, this was a qualitative focus group study. Four focus groups (two in urban areas and one each in rural and semirural areas), consisting of seven or eight occupational therapists with at least three years of relevant practice experience, convened twice to narrate and explore their support of older persons. All were participating voluntarily with confidentiality of their participation being guaranteed by the researchers. They met for a third time to verify emerging analytic results. Data were analysed using a reflective thematic analysis.

**Results:**

Identified were three themes, namely, calling forth powers of occupations, imagining client's future, and cocreating plots, which we synthesized into recurring cocreations from emerging opportunities. *Discussion*. Supporting the resumption of occupations among older persons with physical impairments hinges on repeated processes of identifying possibilities for occupation, followed by actions to bring these (e.g., images of clients' future) into reality. Occupations' healing properties (i.e., occupations' powers) can be used to assist clients in experiencing health and well-being. The results suggest a reframing of occupational therapy practices as recurring processes of recognizing opportunities for occupation, followed by actions whereby these possibilities are turned into reality. Occupational therapy effectiveness might be enhanced when goals and methods are repeatedly and creatively aligned with the evolving plots cocreated between the client, therapist, and stakeholders.

## 1. Introduction

In Japan [1–3] and internationally [4–6], occupational therapy for older adults has predominantly been provided in institutions where the focus of interventions was mainly on remediation of persons' impairments and enabling their self-care performance [1–6]. The more recent practices in clients' home and community environments also necessitate, in addition to supporting older persons' recovery from illness or injury, enabling household chores, leisure, productive endeavours, and community participation, which are also considered important to older persons' daily lives and their health [1, 2, 5–8]. Accordingly, occupational therapists are called upon to place occupation at the core of their role and shift their practice to occupation-centred practices through occupation-based and occupation-focused interventions [1, 2, 8]. Yet, in Japan, occupational therapists supporting older adults with physical impairments report difficulties in responding to this call because medically oriented practice arenas and client preferences for remedial exercises are experienced as a hinder in shifting the foci of their practices towards occupation-centred practices [1–3].

Moreover, Japanese and international research has shown that, particularly for older persons with physical impairments, occupational therapy practice remains overly focused on functional recovery and self-care [1, 2, 9–13]. This study was focused on occupational therapy for older persons with physical impairments as it was part of a research project that aimed to describe and understand how persons from this population resume occupations after illness or accident [14]. Research has identified challenges to implementing occupation-centred practices such as work-place cultures and reimbursement systems emphasizing mitigating impairment, client preferences for recapturing physical functions, and occupational therapists' ambiguous knowledge and attitudes or lack of mutual understanding between clients and occupational therapists on the said practices [9, 15–19]. To understand how occupational therapists deal with such challenging conditions, the focus of this study on occupational therapists in Japan is of relevance, because they work in a country where the greying of society develops ahead of any other [20] and, in Japan, the introduction and development of the profession is intertwined with that of physical therapy and strongly influenced by the medical establishment [1]. Also, to assist occupational therapists to deploy occupation-centred practices [14] in interprofessional contexts and in collaboration with clients, their families, and other relevant stakeholders, the Japanese Association of Occupational Therapists introduced the management tool for daily living performance [2]. This is a practice recording tool that supports identifying clients' occupational needs and planning occupation-centered practices, things hitherto not achieved despite the existence of international models and frameworks that place occupation at the core of the profession. Therefore, important insights can be offered from investigating Japanese occupational therapists' experiences with deploying occupation-centered practices. Accordingly, the aim of this study was at exploring and understanding occupational therapists' experiences of supporting the resumption of occupations among older persons with physical impairments, in Japan.

## 2. Methods

As occupational therapy practices are socially negotiated and constructed, this qualitative research was situated within the constructivist paradigm. Focus groups were used for data gathering [21, 22], as data pertaining socially constructed practices were sought for. In line with the interpretative nature of analysing narratives, reflective thematic analysis was employed to elucidate processes of how participants practiced with older adults with physical impairments [23]. The first author, who did the bulk of the research activities, was a male university faculty in occupational science and therapy with nearly 20 years of experience in doing qualitative research among older adults and occupational therapy students and practitioners. The coauthors were four occupational therapy faculty, a nursing faculty, and a master's degree in occupational therapy student. The four located in Japan assisted in conducting the focus groups, and all coauthors participated in data analysis and writing of this paper.

### 2.1. Participants

Recruitment followed purposive and snowballing sampling methods [21]. To ensure participants' ability to recall and vividly share experiences, inclusion criteria were as follows: occupational therapists currently practicing with older persons and having done so for three or more years. To facilitate variety among participants in terms of years of experience and practice settings, the first author or persons from his networks handed out flyers calling for voluntary participation at local study meetings where such occupational therapists were likely to attend. When responding to emails of applicants, the first author verified that candidates met the inclusion criteria.

Thirty occupational therapists participated, 20 females and 10 males. There were four focus groups consisting of seven or eight participants, which are the appropriate numbers for this kind of study [21]. Participants had 3 to 11 years of relevant experience with a further one having 23 years. They were working in acute care (4), in inpatient rehabilitation (18), as home-visiting therapists (6), in day care (4), and in a nursing care convalescence home (1), and these numbers include four participants who worked in both acute and rehabilitation care. The participants' characteristics reflect national statistics on occupational therapists' gender and years of experience [1, 24, 25]. The first two focus groups were conducted in metropolitan areas, a third focus group in a rural area, and a fourth focus group in a semirural area. To produce transferable analytic results, data from rural and urban areas were aimed for, as in rural areas, traditional multiple generation households are more prevalent than in urban areas, shaping the occupational needs of elderly people.

While some participants had never met, many knew each other from participating in study meetings or being (former) colleagues. Most participants of three of the four focus groups were acquainted to the comoderators. Some had previously interacted with the moderator/first author in occupational therapy study meetings, and two were his former students. As these relationships were 5 to 10 years prior, no conflict of interest was deemed to exist. In the introduction to the focus groups and procedures, the researchers stated that the aim was at learning from their practices and at preventing bias by refraining from referring to the impetus towards occupation-centered practices. Collegial/amicable interactions in the contexts of the focus groups suggested no need for managing power relationships with the researcher or between participants. In five out of eight focus group sessions, one or two participants were absent due to conflicting work schedules.

All were participating voluntarily with confidentiality of their participation being guaranteed by the researchers. Ethical approval was obtained from the local university research ethics board. Participant names in this paper are pseudonyms.

### 2.2. Data-Gathering Methods

Focus groups were conducted employing proceedings and facilitating techniques based on guidelines suggested by Stalmeijer and colleagues [21]. Focus groups were preferred over individual interviews as interactions between participants were considered conducive to exploring a phenomenon that was of a social nature and because focus group interactions were more likely to produce in-depth exploration of their experiences [21, 22]. Accordingly, stories of participants' experiences and reflections thereon were elicited to jointly establish possible meanings that they enacted in their practice [26].

All four focus groups convened twice, spaced by approximately one week, with a third-member-checking meeting to verify emerging analytic results. Three of the focus groups met in a meeting room at a local educational institute, and the rural focus group gathered in a rehabilitation hospital's meeting room. Multiple focus groups also allowed for exploring experiences beyond insights particular to each focus group by sharing insight from the earlier focus group with later groups. This sharing was not done in the first sessions to avoid the risk of leading focus groups into discourses of preceding focus groups. The shared information was also limited to analytic hunches developed from perusing prior focus group transcripts.

The first author moderated the focus groups. He introduced the main questions/topics for discussion and generally led the discussions. The assistant moderators also facilitated participants to explore the presented experiences in depth by prompting participants' reflections on each other's stories. The same process was repeated during the second session, albeit that a handful of topics based on the initial analyses of the first session guided the discussion. The major questions/topics introduced to the participants are outlined in the Appendix. The duration of the focus group discussions ranged from 70 to 100 minutes. The sessions were audio recorded with participant consent.

### 2.3. Data Analysis

Data were analysed using a reflective thematic analysis [23]. The analysis was chosen to generate understandings of the processes of assisting the resumption of occupation among older persons with physical impairments and focused on identifying common experiences and latent meanings. To maintain focus on the process aspect of “supporting the resumption of occupation,” the analysis was guided by constantly posing questions to the data such as “what is going on?” and “how is this unfolding?” The analysis included procedures executed in an iterative, constant-comparative, process described as follows.

The first author carefully read the verbatim transcribed audio recordings, and he verified nuances by listening to these IC recordings. From the data, he identified stories of participants' specific experiences with older persons and noted initial analytic memos. Through repeated perusal of the data, he gained a thorough understanding of the data enabling the coding of meanings contained in chunks of text that signified a process. Examples of codes included the following: change being facilitated, client imagining his/her future, accepting other's reasoning, learning from experience, and sharing understandings for the effective process. As the coding process proceeded, codes were added, merged, and/or divided until a list of codes resulted that provided the best possible illustration of the meanings from the data. Additionally, coauthors read the verbatim transcripts and critically reviewed the codes for each of the focus groups that they had been comoderator for but they did not code themselves. As a way of verifying the quality of analysis afterwards, some minor revisions of coding were indicated to better reflect the meanings in the data. This also indicated that no bias or misunderstandings had influenced the first author's analysis.

In the latter stages of the analysis, identified codes sharing similar meanings were grouped into twelve categories. Following in-depth discussions among the coauthors, they identified several meanings shared across these categories. This resulted in them identifying three themes that best explained the participants' experiences.

Coding and categorizing were supported using ATLAS.ti software, version 7.5.2.

### 2.4. Trustworthiness

Trustworthiness was pursued following common practices for focus group studies [21]. Credibility and confirmability were established by gathering rich data and using the ATLAS.ti memo functions to define codes and to note analytic hunches. Emerging analytic results were refined through discussion among coauthors and through critical review of emerging findings at study meetings of occupational therapy and science scholars, including PhD students, with expertise in qualitative research and the research topic. These meetings also ensured researcher reflexivity and peer debriefing. The final themes were also verified through member checking. Participants confirmed that the analysis reflected their experiences but suggested edits in theme titles to better reflect the language that they had used. For example, a theme tentatively titled “pursuing what matters in occupation” was changed to “calling forth powers of occupations.” Dependability was established when the fourth focus group results indicated that saturation had been met.

## 3. Results

The following three themes were identified: calling forth powers of occupations, imagining client's future, and cocreating plots. The themes were synthesized into the phrase (also used in the title of this paper): reoccurring cocreations from emerging opportunities.

### 3.1. The Three Themes

#### 3.1.1. Calling Forth Powers of Occupations

Participants focused on eliciting potentials embedded in occupations and therapeutic situations. These potentials were to be capitalized upon to create possibilities that could be turned into reality. Mitsuo spoke of “*the powers of occupations*” when responding to other participants talking of how clients, by engaging in occupation as opposed to exercising, gained access to occupations' potentials such as restorative/therapeutic effects, affording self-expression and being recognized in a role, connecting to other people, and facilitating development and change.

Kayako illustrated how a client with rheumatoid arthritis (RA) was able to benefit by calling forth different powers of a craft that she introduced to the client admitted to a long-term care ward in the hospital where she worked.

“*This person, admitted to my hospital, was very introverted… Because of her RA she had gradually become unable to undertake housekeeping and had become a person cared for by her family… I simply considered things she might physically be able to do, given her RA, so proposed to her doing Perler beads*” (Perler beads, also called Hama or Nabbi beads, are plastic colorful beads that can be arranged to form patterns or images and then fused together with an iron for clothes. They can also be strung or woven into necklaces, key chains, etc.).

Kayako reasoned that she intentionally called forth the client's active participation in a craft occupation. Explaining what happened later, Kayako described how her intention was followed by newly emerging powers being turned into reality.

“*She became quite skillful and made one creation after another. Staff and other patients began asking her advice on design and skills or requested her to make things… So, through this occupation another side of this person emerged. From an introverted person she became almost like an instructor!*”In this development, Kayako did not clarify whether she had anticipated these other powers to emerge and be capitalized upon, i.e., developing a new role and connections to other persons that came with the new role. Reflecting on these developments, Kayako and Naoko suggested that it was “*fortuitous*,” suggesting that it was by chance. However, Yumiko and Tsutomu challenged fortuity as playing a role in successfully introducing a craft to this client. They suggested that it had developed more organically by pointing out that creating occupational situations serves to result in discoveries, such as how this occupation's powers facilitated Kayako's client to develop a new role and transform from an introverted to a more sociable person through engaging with other people via the craft. Either way, participants practiced openness for powers of occupation to emerge, then to be recognized and capitalized upon. Hiroko summed up such an experience as “*not just provide a craft, but rather creating a space where it's not known what would be best to arrive at*.” In these multiple ways, powers of occupations were called forth leading to changes, such as developing new skills and creating new roles. This and the following experiences illustrate that occupations' powers could be called forth intentionally, organically, and by chance while engaging clients in evolving occupations.

Mariko, who worked in a nursing home, put forth a more intentional way of calling forth powers of occupation. She told of calling forth healing powers by making use of allegorical aspects of craftwork, cooking, and other occupations. She explained that “*There's an aspect of re-creation after destruction that touches persons' hearts… after all they also have a kind of damage to their body… when making things we damage the original [as with cutting materials in craftwork, cutting vegetables when cooking]… Making a new shape, something with meaning… It links to making a story of recovery, occupations can link to any such story and have this therapeutic effect*.”

In such ways, participants discussed healing powers of occupation being called forth as clients partook in occupation. Participants' also created conditions that led clients to organically benefit from the powers of occupation. For example, Chihiro spoke of creating conditions that would “*activate [a client's] motivation switch*”, explaining about creating the opportunity to care for a plant; “*it's not that [I] moved her heart, but her heart moved (by the client engaging in a personally, meaningful occupation)*”. Utilizing groups was another preferred approach to organically capitalize on powers, which in groups arose from social interactions. For example, socializing among peers as part of occupational therapy was seen motivating clients to engage in occupations and clients could feel that they were needed for others when joining in occupations with their peers. Interestingly, Junko argued that oftentimes, the occupation was of relative importance to clients, as she regarded that the desired effect of socializing could be obtained from “any” occupation. She explained that “*Participation can be around crafts or some exercise, whatever… clients come down to the rehab room, sit down besides whomever and connect… any occupation is good to create that bridging effect*.”

In conclusion, participants and clients called forth powers contained in clients' daily life occupations or in therapeutic situations. They did so by grasping opportunities to capitalize on emerging possibilities and bringing these into reality. Participants achieved this intentionally, when powers were identified as these emerged by chance, and organically by designing situations for powers of occupation to emerge. This afforded clients to benefit in various ways due to the versatility of the occupations in which they engaged.

#### 3.1.2. Imagining Client's Future

Participants used words and expressions like “images” and “imagining the future” when talking about client's future lives. Participants and clients “imagining the client's future” helped to direct occupational therapy practices by raising what issues needed addressing and which of the client's preferences required prioritizing. Furthermore, participants using “*imaginin*g” and “*image of*” a client's future said that often, they and the client themselves were not clear about what clients' daily occupational lives might look like, due to limited knowledge, uncertainty about clients' prospects of recovery, or because changes in clients' conditions made known information less useful. As a result, occupational therapy support was presented as processes of progressing insights into clients' situations evolving from repeatedly revising or concretizing future images and revising goals and support methods accordingly.

Yoko illustrated how this played out by citing the experience with a female client who stated that six weeks into a three-month inpatient rehabilitation period, she was too tired to engage in the prescribed practices, which prioritized self-care and mobility in anticipation of discharge home. First, Yoko explained that the therapy process became void of content because of the client's discontinuation of working on the mutually agreed goals of practicing self-care and mobility skills and improving underlying physical functions. “*One week, two weeks passed, and I started wondering if [the client would acquire the activities of daily living skills] in time for discharge*.” However, Yoko went on to describe how one day, the presence of the client's daughter provided an opportunity for developing alternative and more concrete images together. Yoko said that “*I asked them to tell me what kind of life she had lived before her illness... When [the mother] responded she felt unable to [live like she used to], I thought for the first time she talked about her daily life, and this was a point for me to grasp*.” Yoko identified the first time that the client talked about her daily life as being an opportunity to create images of a possible future, which she facilitated as follows: “*I asked her to write down how she spent a typical day before her illness and now in hospital. When she saw the result, she commented something like ‘oh, I really behave like a sick person.'... So, I asked [the mother and daughter], what kind of daily life would they want [for the client] after discharge?… They responded [the client] used to be outgoing, having fun with friends… They talked among themselves and suggested attending day-service*.” Encouraged to look beyond physical functions, the client realized how she lived her past and current daily life, and from those experiences, the three of them were able to create more concrete images of daily life in the future. Yoko then reported how they then reformulated the occupational therapy goals and program according to the newly developed images.

The abovementioned experience served to illustrate that participants and clients developed images of the clients' future, which could change over time. Other participants shared similar experiences as those highlighted by Yoko and, for the lack of clear future images, particularly in acute and early rehabilitation phases, often resorted to standard practices. These standard practices could be working on self-care and mobility, because “*clients have to live anyway*,” assuming that these are skills indispensable for daily life in the hospital and at home after discharge. However, in contrast to participants working in clients' homes, participants working in rehabilitation hospitals reported that in the beginning of rehabilitation, clients lacked knowledge and experience necessary for imagining their future. In such conditions, clients rather preferred to focus on recovery of physical functions. Participants agreed that “*people anyway would want to recover [physical functions]*” and that such attitudes were reinforced by hospital environments where people focused on “*curing illness*.”

Various approaches as trial and error, taking one thing at a time, and clients' increasing experiences assisted participants and clients in concretizing clients' future lives. Tsutomu reporting experiences of inpatient rehabilitation explained that listening to the clients' stories of “*times when they thrived*” created bases where clients could start imagining what they might want to pursue. Clients' roles and preferences for how they want to live were also featured strongly. Yumiko summed this up as “*it's not just what matches their abilities… it's what suits them*.” Developing images of clients' future was particularly effective when discharge was nearing, “*because clients return to their life… it's the time they begin envisioning daily life*.” Participants described clients' short stay in their homes, as part of preparing for discharge, as “*it raises real daily life issues, experiences, what they want to be able do*.”

Participants regarded practicing of/engaging in occupations gave clients easy to understand feedback on their possibilities for participating in occupations. On the other hand, participants reported struggling for knowledge such as the lack of evidence to inform decisions when safe performance of occupations was in doubt and how to judge the risk of mental stress when matching occupations and clients.

In conclusion, “imagining the client's future” informed and steered processes of resuming occupation. Drawing from past and new experiences, knowledge, and clues in the environment facilitated the discovery and development of images, followed by pursuing the identified possible futures of clients.

#### 3.1.3. Cocreating Plots

Participants stressed the importance of sharing understandings with clients and others for effectively supporting clients' resuming occupation. During a member checking session, Hitoshi termed this “*plots*” to denote that occupational therapy involved schemes of bridging the gap between clients' present and their envisioned future. Participants cocreated plots with clients and other stakeholders that reflected their shared understandings about the directions and methods of clients' resumption of occupations.

Emiko shared her experiences that illustrated the cocreation of one plot from three initially separate plots: one held by her, one held by the client, and another one held by palliative care ward staff. The cocreated plot developed after a male client, with terminal cancer, declined the occupations that Emiko had proposed that he would do as part of his palliative care. Emiko considered the client engaging in his hobby of painting and writing farewell letters as meaningful, but she explained that “*he told me he was not interested in doing his painting and having already completed his farewell letters and greetings*.” Thus, at the start of occupational therapy, Emiko's plot of occupations that she thought as being beneficial did not align with what the client thought would be an occupation beneficial to his well-being. That occupation was his last wish of being able to freely wander around the hospital, as he did around the streets of his downtown neighbourhood. However, that wish was at odds with an institutional plot around risk management that prevented the client from mobilizing independently. In response to the client's wish, Emiko abandoned her idea and explained that “*I proposed to work on his skills for safe mobilizing in a wheelchair and to consult with the ward's palliative care nurse and physician regarding independent mobilizing*.” Following their successful practice of the client's mobilizing skills and Emiko's advocacy on his behalf, permission for “wandering around the hospital” was given. Here, Emiko successfully exploited the acquired mobilizing skills when negotiating on the client's behalf. In conclusion, this experience served to illustrate how participants, clients, and other stakeholders were able to cocreate plots through negotiating and merging perspectives around a meaningful occupation.

Other participants reported too how they likewise endeavoured to merge occupational therapy plots with those of clients. For example, Naoko explained that “*our approaches should not divert from how aged persons wish [daily life] to be. That's our responsibility*.” Participants also applied cocreating plots as a requirement for “*hitting it off together*,” as Makoto put it. Yoko's experience of establishing a mutual understanding and enhancing the clients' motivation to achieve the reaffirmed goals when reassessing a client's occupational needs and preferences together (abovementioned as an illustration of the imagining client's future theme) can also be understood as a cocreation of a new plot.

Evolving insights, e.g., of the elderly client in the abovementioned example and Kayako's experience of the benefits gained by a client from engaging in the craft of Perler beads, illustrate not only that cocreating plots are continuous endeavours but also that cocreating plots are not necessarily put into words and rather are enacted through the experiences with occupation and occupational therapy. Such enacted plots were also used to overcome clients' resistance to discuss needs that participants identified as important, e.g., preparations for daily life after discharge. For example, Hitoshi and Makoto shared how they engaged clients in their private struggles with cooking while exercising clients' physical functions. Their inputs served to raise the clients' interest in teaching cooking skills to their therapists. This resulted in practice situations whereby clients became engaged as cooking instructors to Hitoshi and Makoto in ways that also benefitted their preparations to resume cooking after discharge. This can be seen as these therapists are developing a cocreated plot where the therapist and client plots were integrated through joined actions.

Conversely, participants also reported struggles with sharing their professional intent, as Junko explained that “*I want [the client] to take some things in, as I want her to live life to her fullest*.” However, Junko reported that, because of the client's resistance to discuss practical matters as well as the client's vulnerable mental state, she had refrained from acting on her professional plot and instead had instructed the family on how to ensure cooking safety at home. Other participants too reported on similar struggles with clients whose psychological or cognitive issues constrained their opportunities for cocreating plots.

In conclusion, participants regarded being on the same page with clients and other stakeholders (e.g., family and other care providers) as requisite for success. Plots were cocreated through communicating clients' preferences and professional intent and then further shaped by conditions, images of a client's future, and, last but not least, through the experiences of enacting narratives in daily life and therapeutic situations.

#### 3.1.4. Synthesizing the Three Themes: Reoccurring Cocreations from Emerging Opportunities

During discussions and debriefings, participants remarked how they were learning from the focus groups, particularly that they lacked language to adequately explain their experiences, as one participant said that “*there were things I could organize my thoughts about, but maybe I still don't have the language to clarify*.” Further probing for latent meanings in the data of participants' experiences revealed that much was going on impromptu. For example, powers of occupation were being called forth not only intentionally but also organically or by chance. Evolving insights into clients' future and the repeated cocreation of plots further highlighted occupational therapy as flexible and changeable processes. Synthesizing the three themes, it was observed that cocreations began with recognizing opportunities, which were then followed by actions of occupational therapists and their clients whereby possibilities (i.e., occupations' powers or images of clients' future) were turned into reality. Accordingly, this overarching theme was labelled as follows: reoccurring cocreations from emerging opportunities.

## 4. Discussion

Before discussing the results, it must be acknowledged that participants told of pursuing plans of remediation of functional impairments, of skill acquisition, and/or of modifications in the environment and other adaptations. In this paper, these are not presented as such approaches are extensively covered in international occupational therapy literature. Rather, the phrase “reoccurring cocreations from emerging opportunities” was put forth as explicating the new knowledge of supporting older persons. The phrase also provides a vocabulary for explaining occupation-centered [14] occupational therapy.

The theme of calling forth powers of occupations is in line with concepts of potentiality [27] which is relevant in understanding an individual's future possibilities for participating in occupations. The authors redefined potential as also a latent possibility to act in occupations, as if occupations invite people to act and benefit of the occupational experience. Thus, capitalizing on emerging occupational powers (potentials) not only pertains to aligning occupations and a person's capacities but also to providing (older) clients with experiences of health through participating in occupations. This is what the participants in this study meant when they spoke of powers, such as connecting to other people, being afforded self-expression, and being recognized in a role.

This raises the question, which seems worthwhile to be studied further, whether occupational therapists, internationally and in Japan, consider health not only from a capacity for engaging in occupations but also from a perspective of ageing with dignity by leading daily lives according to people's preferences and abilities [20, 28]. Accordingly, this theme resonates the notion that finding meaning in occupations of daily living is important to health [29, 30]. Nevertheless, these interpretations of the findings lend further support to the notion that participating in occupations can afford experiences of health, irrespective of older persons' capabilities to perform occupations or their status after incurring a disabling illness or injury [31].

The second theme (imagining client's future) shows that images of client's future can be fluid and often not clear at all. Indeed, the examples of Kayako and Yoko challenge the idea of occupational therapy as predictable processes, be they represented as linear, circular, or spiral [32]. The findings show that occupations to be pursued might not be easily identified and turned into goals to be achieved. Rather, occupational needs and preferences can change or emerge according to clients' evolving situations. An earlier study among elderly persons with physical impairments similarly concluded a judicious use of different approaches and warned against goals and treatment plans set in stone [31]. From a narrative perspective, this is in line with Josephsson and colleagues who argue that engaging in occupations creates situations for creatively exploring possibilities and meaning making [33]. Applying an understanding of transactional theory to engaging in occupation [32] similarly favours a more fluid ends-in-view approach instead of setting long-term goals in stone.

The theme of cocreating plots aligns to the idea of occupational therapy as emergent and enacted narratives [26]. As an emergent plot, how cocreation might be achieved was not fleshed out in detail in this study, but Shimada shows the dynamics of differing perspectives that occupational therapists and clients bring into their evolving and eventually ending relationship [34]. Others show, similarly to this study, that cocreation is facilitated by flexibly and mutually adjusting goals and methods, as facilitated by sharing clients' experiences of participating in occupation [35]. Further study on this dynamic seems important to advance client-centred and occupation-centred practices.

Finally, the overarching theme of cocreation from emerging opportunities can be understood as providing a vocabulary that the participants were lacking to fully articulate how they performed occupational therapy. This raises the questions, for further study, whether current professional discourses fall short of fully explaining how occupational therapists support older clients and/or whether professional language not quite suits Japanese sociocultural contexts [1, 36]. Nevertheless, it would seem worthwhile that the themes are adopted to explain occupational therapy.

### 4.1. Implications for Practice

The “impromptuness” identified in this study cautions against determining occupations that should be subject of occupational therapy, either at the outset of treatment or even at set intervals. Instead, an on-going process of assessing and verifying the client's situation is advised as clients' occupations and their meanings are not stable entities but evolve. This also implies that plans are liable to becoming redundant somewhere along the way of clients resuming their daily lives. Constantly cocreating plots would also serve to attune professional approaches to clients' evolving situations.

Benefitting from being open and flexible, to capitalize on newly emerging opportunities instead of rigidly adhering to set goals and plans to achieve those goals, would enhance occupational therapy's efficacy. Instead, occupational therapists should be open minded to twists and turns. As well, they should be open minded to the possibility that needs or preferences, goals, and plans emerge and wane with their own beginning and ends [31, 35], some intentional and other by chance [35].

Furthermore, thinking of therapeutic processes as drawing from occupational powers can prevent three risks. First, calling forth occupations' healing powers, e.g., rejuvenating experiences and fulfilling a social role, can enhance clients' experiences of health. This can be particularly important for those people who have limited possibilities for recovery of impaired functions. This will also contribute to preventing the risk of holding clients responsible for not achieving their potential based on narrow perspectives of individual's (latent) abilities [27, 37]. This can also be relevant for older persons who are restricted by barriers in their environment or whose values lead them to choose differently than what is commonly considered “good,” for example, because they lack vigor for engaging in occupations or rehabilitative efforts [38]. Third, pursuing long-term goals might run the risk of putting clients' health on hold until achieved. Instead, health can be promoted by drawing on powers of occupation, even when older persons are still recovering from disabling illness or injury [31].

### 4.2. Methodological Considerations

This study tapped into narrative functions of giving meaning to experiences and gaining insights into occupational therapists' thoughts and actions [26, 39]. Participants' reflections about learning from the focus groups and them expanding on each other's stories are in line with the stated benefits of focus groups [21]. In this sense, participants not merely communicated their experiences but constructed and reconstructed these [26, 39]. While the three themes clearly resulted from the reflective thematic analysis, the phrase “reoccurring cocreations from emerging opportunities” can be seen as the result of emplotting these three themes [26, 39].

Given the geographic spread and variety of participants' characteristics, the finding might be seen as representative of occupational therapists who work with elderly persons with physical impairments but might need confirmation with those working on Japan's remote islands and (depopulating) rural areas. Furthermore, the experiences shared were told as filtered through participants' memories, which can be more or less clear. Furthermore, it cannot be excluded that their moral sensitivities and interactions in the focus groups limited participants in sharing certain experiences and opinions. Accordingly, more study is warranted, for example, through (participant) observation studies of real-life occupations and occupational therapy situations. Studies like this by other researchers and among different groups of occupational therapists should confirm, refute, and/or refine the themes identified from this analysis [26].

## 5. Conclusion

The three themes illustrate that supporting the resumption of occupation among older persons with physical impairments involves unfolding, recurrent processes. Creating possibilities was central to resuming occupation through acting on powers of occupation emerging from occupational therapy and daily life situations. Based on repeatedly recognizing and acting upon these emerging powers, creating possibilities can be at the core of resuming occupation and affording older clients to experience health. Cocreating and enacting shared plots can serve to creatively and iteratively employ different approaches that match changing preferences, needs, and conditions of older persons.

## Data Availability

Access to raw and processed data is restricted due to ethical regulations.

## Appendix

### A.1. Outline of Focus Group Proceedings

#### A.1.1. Introduction (All Focus Groups' First Session)

An explanation of the research focus of exploring how elderly persons with physical disabilities resume occupations after illness or accident is discussed, followed by an ice-breaker exercise.

#### A.1.2. Starting Question

“The interest is in stories that relate to events and experiences whilst working with older clients with physical disabilities, particularly how these relate to these clients resuming their occupations or daily lives. These stories may describe events evolving over an extended period or be related to a particular episode. The stories may be about positive or not so positive experience that occurred in hospital, clients' homes, or in the community.”

#### A.1.3. Introduction to the Second Session for Each Focus Group

After reiterating the group focus on resumption of occupation and verifying a short summary of the discussions in the first session of the focus group, the topics for the second session were as follows:

##### A.1.3.1. 2^nd^ Session Kanto/Tokyo (Urban) Focus Group

What do you think about how older clients perceived/experienced their changes? What meaning did clients give to their life stories in their readjustment to daily life? What types of lifestyle would you consider older clients prefer?

##### A.1.3.2. 2^nd^ Session Kansai/Kobe (Urban) Focus Group

Please, discuss dilemmas of training functions instead of practicing occupations, such as activities of daily living, particularly in relation to preparing for discharge. Please, discuss examples of positive or negative outcomes when using different approaches. In reference to the Kanto group, did they experience tensions around their (preferred) practice not being recognized by institutional/health care system policy? What do you think about how older clients perceived/experienced their changes? What type of lifestyle would you consider older clients prefer?

##### A.1.3.3. 2^nd^ Session Kansai (Rural) Focus Group

From your clients' point of view, what might be a good daily life for older persons? Please share stories of change as older clients resume their daily lives, like during hospitalization, and after discharge. About the impact of environment and involving staff on goals and methods, please share examples of effective or not so effective experiences. How do you use the power of occupation (for their older clients)? Please share stories about experiencing really feeling the power of occupational therapy.

##### A.1.3.4. 2^nd^ Session Aichi (Semirural) Focus Group

Please share stories about different kinds of change in older clients and how you supported. Please share experiences about making use of the power of occupation. Sometimes, one-on-one support was not so effective as compared to approaching the environment and collaboration with other professions: please share examples of effective or not so effective experiences. Seen from older clients' point of view, what is probably a good life?
